# Fuzzy C-Means Algorithm-Based ARM-Linux-Embedded System Combined with Magnetic Resonance Imaging for Progression Prediction of Brain Tumors

**DOI:** 10.1155/2022/4224749

**Published:** 2022-03-15

**Authors:** Haibo Wang, Tieshi Song, Liying Wang, Lei Yan, Lei Han

**Affiliations:** ^1^Center of Modern Educational Technology, Mudanjiang Medical University, Mudanjiang, 157011 Heilongjiang, China; ^2^Information Center Hongqi Hospital Affiliated to Mudanjiang Medical University, Mudanjiang, 157011 Heilongjiang, China; ^3^General Services Branch, The Second Affiliated Hospital of Mudanjiang Medical University, Mudanjiang, 157009 Heilongjiang, China; ^4^Department of Histology and Embryology, Mudanjiang Medical University, Mudanjiang, 157011 Heilongjiang, China; ^5^Information Section, The Second Affiliated Hospital of Mudanjiang Medical University, Mudanjiang, 157009 Heilongjiang, China

## Abstract

The aim of this research was to analyze the application of fuzzy C-means (FCM) algorithm-based ARM-Linux-embedded system in magnetic resonance imaging (MRI) images for prediction of brain tumors. The optimized FCM (OFCM) algorithm was proposed based on kernel function, and the ARM-Linux-embedded imaging system was designed under ARM9 chip and Linux recorder, which were applied in MRI images of brain tumor patients. It was found that the sensitivity, specificity, and accuracy of the OFCM algorithm (90.46%, 88.97%, and 97.46%) were greater obviously than those of the deterministic C-means clustering algorithm (80.38%, 77.98%, and 85.24%) and the traditional FCM algorithm (83.26%, 79.56%, and 86.45%), and the difference was statistically substantial (*P* < 0.05). The ME and running time of the OFCM algorithm decreased sharply in contrast to those of the deterministic C-means clustering algorithm and the traditional FCM algorithm (*P* < 0.05). There were great differences in fraction anisotropy (FA) and mean diffusion (MD) of tumor parenchymal area, surrounding edema area, and normal white matter area (*P* < 0.05). FA of stage III+IV was smaller than those of stage I and II (*P* < 0.05), while the apparent diffusion coefficient (ADC) of stage III+IV was greater than that of stage I and II (*P* < 0.05). In conclusion, the poor update data processing and low data clustering efficiency of FCM were solved by OFCM. Moreover, computational efficiency of ARM-Linux-embedded imaging system was improved, so as to better realize the prediction of brain tumor patients through ARM-Linux-embedded system based on adaptive FCM incremental clustering algorithm.

## 1. Introduction

Brain tumors are all kinds of intracranial tumors, which can be divided into benign and malignant tumors. The growth rate of benign tumors is relatively slow, and the body surface is relatively smooth. In most cases, brain tumors can be completely removed by surgery, and the good therapeutic effects are achieved [1, 2]. Most patients with brain tumors rarely relapse after undergoing surgeries. Even if there is a recurrence, surgery can be considered again. Malignant tumors tend to grow faster, easily adhere to surrounding tissues, and are difficult to achieve the complete surgical resection. Besides, they are prone to recurrence after surgery and distant metastasis and cause invasions to the surrounding brain tissues, blood vessels, and nerves, resulting in serious neurological dysfunction [3]. There are many types of brain tumors, among which benign brain tumors generally include meningioma, schwannoma, and pituitary tumors, while malignant brain tumors commonly include oligodendroglioma, ependymoma, and medulloblastoma [4, 5]. Unfortunately, the cause of brain tumors is still unclear. It is generally believed that the occurrence of brain tumors is related to oncogene mutations. Some oncogenes occur on germ cells and will be passed on to the next generation [6]. When the volume of brain tumor is small at the early stage, the patient has no obvious clinical symptoms. When the volume is large, symptoms of severe intracranial pressure will be increased, such as severe headache, nausea, vomiting, and even disturbance of consciousness and confusion. Therefore, how to detect and treat brain tumors early is the focus of current clinical research. MRI is a medical imaging technology applied in radiology. It can apply strong magnetic fields, magnetic field gradients, and radio waves to form images of anatomy and physiological processes of the body, without involving adverse factors such as ionizing radiation [7]. MRI-based nuclear medicine imaging systems are extensively used in clinical disease diagnosis. Nuclear medicine imaging systems often have the characteristics of complex system structure and dense local connections. In order to ensure the safety of nuclear medicine imaging systems, it is generally necessary to use special recorders for nuclear medicine imaging system equipment for real-time monitoring [8, 9]. However, the current research and development of nuclear medicine imaging systems are mainly focused on system equipment, and the research on their recorders is rarely involved. Therefore, the objective of this study aimed at the nuclear medicine imaging system to develop its dedicated recorder, so as to provide strong support for the better development, promotion, and application of such systems [10]. FCM algorithm is a clustering algorithm based on partition. Its idea is to maximize the similarity between objects that are divided into the same cluster, while the similarity between different clusters is the smallest. It has been widely applied in automatic image segmentation [11]. Thus, a new automatic image segmentation algorithm was constructed in this study based on the FCM algorithm, which was adopted in the nuclear medicine imaging system. To sum up, nuclear medicine imaging systems are extensively adopted in the medical field, and excellent image processing algorithms are also an extremely critical part. Based on this, the kernel function and the traditional FCM algorithm were first introduced in this study to construct an adaptive incremental image segmentation algorithm, and an ARM-Linux-embedded MRI system was also designed through the ARM9 chip and Linux recorder. This algorithm was compared with the HCM algorithm and the traditional FCM algorithm, and the ARM-Linux-embedded MRI system was applied to the MRI images of patients with glioma to comprehensively evaluate the predictive value of the ARM-Linux-embedded system combined with MRI images in the progression of patients with brain tumors.

## 2. Materials and Methods

### 2.1. Selection of Research Samples

In this research, 110 patients with glioma were selected as research objects, who were admitted to the hospital from March 10, 2017, to May 20, 2020. There were 67 males and 43 females, aged 20-71 years. This study had been approved by the Ethics Committee of hospital, and the patients and their family members had understood the situation of this study and signed the informed consent forms.

The criteria for inclusion were defined to include patients who were diagnosed as brain tumors through clinical pathology, were not received drug treatment, had clear consciousness and were able to cooperate with examinations, and had complete clinical data.

The criteria for exclusion were defined to include patients who suffered from mental illness, had other malignant tumors, withdrew from the experiment due to their own reasons, and did not sign informed consent forms.

### 2.2. MRI Imaging Examination

In this study, 3.0 T superconducting magnetic resonance scanner and 8-channel head coil were employed to scan and examine the patients. Before scanning, they should not eat and drink for 8 hours and had the breathing training. At the beginning of scanning, every patient should be placed in a supine position, and a sponge filling was used to fix the research object's head in order to avoid the influence caused by moving. The scanning parameters were as follows. The matrix was 521 × 521, the layer thickness was 5.5 m, the layer spacing was 1.5 mm, the field of view was 25 × 25 cm, the time of repetition (TR) was 500 ms, and the time of echo (TE) was 40 ms. After the scanning was completed, the image was sent to the workstation for image reconstruction and diagnostic analysis. The largest level of the lesion signal was selected, and the region of interest (ROI) was selected in the lesion, so as to measure the patient's lesion distribution position and different sequence signal types and calculate the diagnostic accuracy rate. The tumor parenchyma area, peritumoral edema area, and normal brain tissue area of the patient were diagnosed by two senior physicians. ROI was selected from each area, and ADC and FA were determined. The FA map, color tensor map, and white matter fiber map were observed in different periods in order to judge the influence of the tumor on the adjacent white matter fiber tracts according to the changes in the position and direction of the fiber bundles. In addition, the influences were mainly divided into no obvious change, movement, infiltration, and destruction.

### 2.3. Adaptive Incremental Image Automatic Segmentation Algorithm Based on FCM

The main idea of FCM algorithm was to find the membership matrix and cluster at this time by satisfying the objective function to minimize the value, thus determining the object's attribution problem by the size of the membership. In this algorithm, the sum of all elements in the membership matrix was 1, which could be expressed as follows.

(1) $$\begin{array}{c} \overset{l}{\underset{i=1}{\sum }}\theta_{ij}=1, \end{array}$$

(2) $$\begin{array}{c} Y=\left\{y_{i},i=1,2,\cdots ,m\right\}. \end{array}$$

In equations (1) and (2), *l* represented the number of cluster classifications, *j* = 1, 2, ⋯, *m*, and *Y* was the set of elements for clustering. Then, the objective function of FCM was shown in the following.

(3) $$\begin{array}{c} P\left(W,l_{1},\cdots ,l_{l}\right)=\overset{l}{\underset{i=1}{\sum }}\overset{m}{\underset{j=1}{\sum }}{w_{ij}}^{n}{c_{ij}}^{2}. \end{array}$$

In equation (3), *w*_*ij*_ stood for the membership degree of the *j*-th element to the *i*-th cluster center, *l*_*i*_ represented the *i*-th cluster center, *P*(*W*, *l*_1_, ⋯, *l*_*l*_) meant the objective function of FCM, and *W* represented the membership matrix. Then, Euclidean distance and weighted index *n* were introduced to optimize the objective function as follows.

(4) $$\begin{array}{c} P^{*}\left(W,l_{1},\cdots ,l_{l},\alpha_{1},\cdots \alpha_{m}\right)=\overset{l}{\underset{i=1}{\sum }}\overset{m}{\underset{j=1}{\sum }}{w_{ij}}^{n}{c_{ij}}^{2}+\overset{m}{\underset{j=1}{\sum }}\alpha_{j}\left(\overset{l}{\underset{i=1}{\sum }}w_{ij}-1\right). \end{array}$$

In equation (4), *α* stood for the Euclidean distance coefficient. Besides, equation (4) was derived to obtain the optimal solution of each variable of the objective function, which was expressed in equations (5) and (6).

(5) $$\begin{array}{c} l_{i}=\frac{\sum_{j=1}^{m}{w_{ij}}^{n}x_{j}}{\sum_{j=1}^{n}{w_{ij}}^{m}}, \end{array}$$

(6) $$\begin{array}{c} w_{ij}=\frac{1}{\sum_{b=1}^{l}{\left(c_{ij}/c_{bj}\right)}^{2/n-1}}. \end{array}$$

Considering that FCM is an unsupervised algorithm, different initial cluster centers need to be confirmed, which affect the image segmentation effect. Therefore, the kernel function [12] was introduced in this study to convert the data in the low-dimensional feature space to the high-dimensional feature space, which could be expressed as follows.

(7) $$\begin{array}{c} \Phi :z⟶U\left(z\in R^{i}⟶\Phi \left(z\right)\in R^{j}\right). \end{array}$$

In equation (7), *Φ* was the nonlinear mapping, *U* stood for the high-dimensional feature space, and *z* represented the low-dimensional feature space. Then, the cluster centers in the high-dimensional space could be shown in the following.

(8) $$\begin{array}{c} l_{i}=\overset{m}{\underset{j=1}{\sum }}\kappa_{ij}\Phi \left(x_{j}\right). \end{array}$$

In equation (8), *κ* meant the low-dimensional feature space data. In addition, the improved FCM objective function could be expressed as follows.

(9) PnW,l=PnW,κ1,⋯κl=∑i=1l∑j=1mwijncijnΦxj−∑l=1mκΦilxl2,

(10) $$\begin{array}{c} l_{i}=\overset{m}{\underset{j=1}{\sum }}\kappa_{ij}\Phi \left(x_{j}\right). \end{array}$$

Equation (9) was the objective function obtained by the inner product operation, and then, the kernel function was introduced to replace the inner product for calculation to realize the mapping from low-dimensional space to high-dimensional space. Thus, equation (11) could be obtained.

(11) $$\begin{array}{c} P_{n}\left(W,\kappa_{1},\cdots \kappa_{l}\right)=\overset{l}{\underset{i=1}{\sum }}\overset{m}{\underset{j=1}{\sum }}{w_{ij}}^{n}\left(T_{jj}-2{\kappa_{i}}^{T}T_{j}+{\kappa_{i}}^{T}T\kappa_{j}\right). \end{array}$$

Next, equation (10) was solved to get equations (12) and (13).

(12) $$\begin{array}{c} w_{ij}=\frac{{\left(1/\left(T_{jj}-2{\kappa_{i}}^{T}T_{j}+{\kappa_{i}}^{T}T\kappa \right)\right)}^{1/n-1}}{\sum_{j=1}^{l}{\left(T_{jj}-2{\kappa_{i}}^{T}T_{j}+{\kappa_{i}}^{T}T\kappa \right)}^{1/n-1}}, \end{array}$$

(13) $$\begin{array}{c} \kappa_{i}=\frac{\sum_{j=1}^{m}{w_{ij}}^{n}T^{-1}T_{j}}{\sum_{j=1}^{m}{w_{ij}}^{n}}. \end{array}$$

Therefore, the optimal solution for each variable of the objective function could be obtained. The above was the optimized adaptive incremental FCM algorithm, denoted as OFCM. The specific process is shown in Figure 1.

### 2.4. Design of Nuclear Imaging System Based on ARM-Linux-Embedded System

The core board+backplane structure was applied to design the main control system unit of the nuclear imaging platform. The core board was mainly composed of ARM, FLASH, power supply, and clock, while the backplane was the various interfaces required by the core board, such as network port, SD port, USB port, and LCD screen.

As shown in Figure 2, the Samsung ARM920T chip S3C2440A was used as the core processor of the nuclear imaging platform, with a main frequency of 400 MHz. The system memory is connected in parallel by two external K4S561632N, forming a 32-bit bus data width with a capacity of 64 MB. The model K9F2G08 of Nand Flash was selected for data storage and processing, with a capacity of 256 MB. Furthermore, 12 MHz passive crystal oscillator was adopted as the system clock.

As for the backplane (Figure 3), the DM9000 network card chip was used as the network port, which could adapt to a 100 M network, and the coupling coil can be connected to the computer with a common network cable. There were two USB interfaces. One was USB host, which could be connected to external storage devices such as U disks for the storage and backup of recorder data. The other was a USB device, which was employed to download programs to the target board to facilitate the debugging of the recorder. The SD end applied the chip S3C2440A integrated SD card interface protocol, which could directly connect to the S3C2440A chip to store related measurement data. The LCD screen adopted a 4-wire resistive LCD touch screen (NL2432HC22), which was mainly used to realize human-computer interaction, thereby obtaining a more intuitive display effect.

Considering that the hardware resources of the embedded system were limited relatively, there were problems such as low frequency, small memory, and no large display. A cross-development environment was built in order to compile a program on the computer platform that can be executed on the hardware platform of the recorder. The hardware environment included recorder, computer, network cable, serial cable, connection cable, and 5 V power supply. What is more, the software environment contained computer Fedora 9 (NFS/TFTP) service, ARM-Linux-gcc 4.4.3 tool chain, and terminal. The design of the embedded Linux system, as shown in Figure 4, mainly included the system boot program (to start the Linux system), the startup parameter area (to store the parameters for system startup), the Linux kernel and drivers, the file system (to provide configuration files), and user application (custom program). Therefore, the recorder based on the embedded ARM-Linux system was designed and applied to the nuclear imaging system.

### 2.5. Algorithm Evaluation Indicators

The deterministic C-means clustering algorithm [13] and the traditional FCM algorithm [14] were introduced to compare with the OFCM algorithm constructed in this study. Misclassified error (ME), accuracy rate, sensitivity, specificity, and running time were selected as evaluation indicators of algorithm performance, and their calculation methods were as follows.

(14) $$\begin{array}{c} \text{ME}=\frac{\text{Area}\left(T_{1}\cup T_{2}\right)-\text{Area}\left(T_{1}\cap T_{2}\right)}{\text{Area}\left(T_{2}\right)}, \end{array}$$

(15) $$\begin{array}{c} \text{Accuracy}=\frac{F_{\text{True}}}{\text{Total}}\times 100\%, \end{array}$$

(16) $$\begin{array}{c} \text{Sensitivity}=\frac{\text{TP}}{\left(\text{TP}+\text{FN}\right)}\times 100\%, \end{array}$$

(17) $$\begin{array}{c} \text{Specificity}=\frac{\text{TN}}{\left(\text{TN}+\text{FP}\right)}\times 100\%. \end{array}$$

In equations (14), (15), (16), and (17), *F*_True_ represented the number of cases with correct prediction, Total expressed the total number of cases, TP stood for true positive, TN represented true negative, FP meant false positive, and FN expressed false negative. What is more, *T*_1_ stood for the algorithm segmentation of the target area and *T*_2_ meant the manual segmentation of the target area.

### 2.6. Observation Indicators

The age, course of disease, gender, and MRI imaging data of patients should be recorded, as well as the FA and ADC values of the tumor parenchyma, peritumoral edema area, and normal brain tissue area. The patients with glioma were staged pathologically based on the central nervous system (CNS) tumor classification method by the World Health Organization (WHO), including stage I, stage II, stage III, and stage IV [15].

### 2.7. Statistical Methods

The data processing in this study was analyzed by SPSS19.0 version statistical software, the measurement data was expressed as mean ± standard deviation ($\bar{x}\pm s$), and the count data was represented by percentage (%). Besides, *P* < 0.05 indicated that the difference was statistically substantial.

## 3. Results

### 3.1. Comparison on the Performance of the Three Algorithms

Figure 5 indicates the comparison results of the sensitivity, specificity, and accuracy of the three algorithms. The sensitivity, specificity, and accuracy of the OFCM algorithm (90.46%, 88.97%, and 97.46%) were greater obviously than those of the deterministic C-means clustering algorithm (80.38%, 77.98%, and 85.24%) and the traditional FCM algorithm (83.26%, 79.56%, and 86.45%), and the difference was statistically substantial (*P* < 0.05). Figures 6 and 7 show the comparison results of running time and ME of the three algorithms, respectively. It was found that the ME and running time of the OFCM algorithm decreased sharply in contrast to those of the deterministic C-means clustering algorithm and the traditional FCM algorithm (*P* < 0.05).

### 3.2. Brain MRI Imaging Manifestations of Some Patients

Figure 8 is a brain MRI image of a male patient (52 years old). It indicated that there were a wide range of diffuse lesions in the cerebral hemispheres, unclear borders of gray and white matter, and inconspicuous space occupation, often involving the corpus callosum and basal ganglia. In addition, there was no enhancement or slight enhancement of MRI and nonuniformity and multifocal enhancement at the progressive stage.  Figure 9 shows a brain MRI image of a female patient (48 years old). The tumor often involved 2-3 brain lobes, the white matter changed mainly, the space-occupying effect was not obvious or there was a slight space-occupying effect, the brain structure of the diseased area was relatively retained, and there was usually no enhancement after enhancement.

### 3.3. Comparison on ADC Values in Tumor Parenchyma Area, Peritumoral Edema Area, and Normal Brain Tissue Area

Figure 10 shows the comparison results of ADC values in the tumor parenchyma, peritumoral edema area, and normal brain tissue area. The ADC value of the tumor parenchyma was greater dramatically than the value of peritumoral edema area and the normal brain tissue area, with a statistically obvious difference (*P* < 0.05). Moreover, the ADC value of the peritumoral edema area increased markedly in contrast to the value of the normal brain tissue area (*P* < 0.05).

### 3.4. Comparison on FA Values of Tumor Parenchyma Area, Peritumoral Edema Area, and Normal Brain Tissue Area

The FA values of the tumor parenchyma, peritumoral edema area, and normal brain tissue area were compared, and the comparison results are shown in Figure 11. It was found that the FA value of the tumor parenchyma was steeply smaller than the value of peritumoral edema area and the normal brain tissue area (*P* < 0.05). Besides, the FA value of the peritumoral edema area reduced obviously in contrast to that of the normal brain tissue area, and there was a statistically great difference (*P* < 0.05).

### 3.5. Comparison on ADC and FA Values of Tumor Parenchymal Area at Different Stages

The ADC and FA values of tumor parenchymal area were compared at different stages, as shown in Figure 12. It showed that the FA value of stage III+IV was lower steeply than that of stage I and stage I (*P* < 0.05), and the FA value of stage II dropped sharply in contrast to the value of stage I (*P* < 0.05). The ADC value of stage III+IV was greater substantially than that of stage I and II, and the difference was statistically significant (*P* < 0.05). What is more, the ADC value of stage II was greater markedly than that of stage I (*P* < 0.05).

## 4. Discussion

At present, MRI is often applied to diagnose brain gliomas in clinics, but routine MRI is easily interfered by the spatial changes of in vivo magnetic susceptibility, which affects the normal presentation of images and delays the diagnosis of physicians. Comparing the algorithm in this study with the deterministic C-means clustering algorithm and the traditional FCM algorithm, it was found that the sensitivity, specificity, and accuracy of the OFCM algorithm were greater hugely than that of the deterministic C-means clustering algorithm and the traditional FCM algorithm (*P* < 0.05). Besides, it revealed that the OFCM algorithm could effectively improve the diagnosis of brain tumors. Moreover, the ME and running time of the OFCM algorithm reduced sharply in contrast to those of the deterministic C-means clustering algorithm and the traditional FCM algorithm, and the difference was statistically great (*P* < 0.05). This was similar to the research results of Su et al. [16], indicating that the OFCM algorithm could not only improve the accuracy of the diagnosis of brain tumors but also shorten the running time of the system, so as to enhance the diagnosis efficiency. The ARM-Linux-embedded MRI system based on OFCM algorithm was applied to MRI images of patients with glioma. It was found that the ADC value of the tumor parenchyma area was greater markedly than the value of peritumoral edema area and the normal brain tissue area, and the ADC value of the peritumoral edema area rose greatly compared with the normal brain tissue area (*P* < 0.05). This was different from the results of Khashbat et al. [17], suggesting that the tumor destroyed the normal nerve fiber myelin structure and caused an increase in extracellular free water. The FA value of the tumor parenchyma area was sharply lower than that of the peritumoral edema area and normal brain tissue area, and the FA value of the peritumoral edema area decreased hugely in contrast to the value of the normal brain tissue area (*P* < 0.05). The FA value could be adopted to evaluate the degree of invasion and infiltration of glioma to the surrounding brain white matter. When tumor cells damage the nerve fiber myelin structure, the FA value will decrease, indicating that the more intense the pressure of glioma cells on the nerve fiber bundles in the brain, the smaller the FA value over time [18]. The FA value of stage III+IV was extremely smaller than that of stage I and II, and the FA value of stage II was steeply smaller than that of stage I, and the ADC value was just the opposite (*P* < 0.05). It disclosed that the damage to invasion and infiltration and the white matter invasion were deeper with the development of glioma.

## 5. Conclusion

The kernel function and traditional FCM algorithm were first introduced to construct the adaptive incremental image automatic segmentation algorithm, and the ARM-Linux-embedded MRI system was designed through ARM9 chip and Linux recorder. This algorithm constructed in this study was compared with the deterministic C-means algorithm and traditional FCM algorithm. What is more, the ARM-Linux-embedded MRI system was applied to MRI images of patients with glioma. It was found that the OFCM algorithm based on the kernel function and FCM algorithm in this study could not only promote the diagnosis accuracy of brain tumors but also shorten the running time of the system, thus improving the diagnosis efficiency. The ARM-Linux-embedded MRI system based on the OFCM algorithm could effectively display the damage of glioma to the nerve fiber myelin structure and the degree of invasion of the brain white matter. It could better predict brain tumors and had certain clinical application prospect. However, there are still some shortcomings in this study. The ARM-Linux-embedded MRI system is still in the preliminary application stage and lacks more detailed functions. In the future, the sample size of patients should be increased, and the nuclear imaging system needs to be perfected, so as to analyze the MRI imaging characteristics of brain tumors. In short, the research results of this study provide a theoretical basis for the application of ARM-Linux-embedded system based on FCM algorithm in clinical tumor diagnosis.

## Figures and Tables

**Figure 1:** Flow chart of the improved adaptive incremental FCM algorithm.

**Figure 2:** Design of the core board.

**Figure 3:** Design of the backplane.

**Figure 4:** Design of the embedded Linux system.

**Figure 5:** Comparison on accuracy, sensitivity, and specificity of the three algorithms. ∗ meant that the difference was statistically obvious compared with the OFCM algorithm (*P* < 0.05).

**Figure 6:** Comparison on the running time of the three algorithms. ∗ indicated that the difference was statistically marked in contrast to the OFCM algorithm (*P* < 0.05).

**Figure 7:** Comparison on ME of the three algorithms. ∗ showed that there was a statistically substantial difference in contrast to the OFCM algorithm (*P* < 0.05).

**Figure 8:** A brain MRI image of one male patient (62 years old) (the blue arrow marked the part of the lesion).

**Figure 9:** A brain MRI image of one female patient (48 years old) (the blue arrow marked the part of the lesion).

**Figure 10:** Comparison on ADC values of tumor parenchymal area, peritumoral edema area, and normal brain tissue area. 1, 2, and 3 stood for the tumor parenchymal area, the peritumoral edema area, and the normal brain tissue area in turn. ∗ meant that the difference was statistically substantial compared with the tumor parenchyma (*P* < 0.05); # indicated that the difference was statistically obvious in contrast to the peritumoral edema area (*P* < 0.05).

**Figure 11:** Comparison on FA values of tumor parenchymal area, peritumoral edema area, and normal brain tissue area. 1, 2, and 3 stood for the tumor parenchymal area, the peritumoral edema area, and the normal brain tissue area in turn. ∗ meant that the difference was statistically substantial compared with the tumor parenchyma area (*P* < 0.05); # indicated that the difference was statistically obvious in contrast to the peritumoral edema area (*P* < 0.05).

**Figure 12:** Comparison on ADC and FA values of tumor parenchymal area at the four stages. ∗ showed that the difference was statistically marked compared with the stage III+IV (*P* < 0.05); # indicated that the difference was statistically obvious in contrast to the stage II (*P* < 0.05).

## Data Availability

The data used to support the findings of this study are available from the corresponding author upon request.
